# Combined Application of CT Perfusion Imaging and CT Angiography in Imaging Diagnosis of Acute Cerebrovascular Diseases

This article has been retracted.

**DOI:** 10.1155/2021/4825285

**Published:** 2021-10-29

**Authors:** Yanjiao Li, Zhipeng Liu, Baojin Wu, Jingrui Zhang, Chao Li

**Affiliations:** Dept Med Image, Heilongjiang Provincial Hospital, Harbin 150036, Heilongjiang, China

## Abstract

The incidence rate of cerebrovascular diseases is increasing year by year, but the accuracy of clinical diagnosis is not high enough to cause disease. Many patients cannot effectively diagnose and treat the disease at the early stage. CT perfusion imaging (CTP) and CT angiography (CTA) were used to diagnose cerebrovascular diseases. In this paper, 26 cases of patients with acute cerebrovascular disease in our hospital from June to August 2020 were selected as the research objects. According to the diagnosis method voluntarily chosen by patients, 6 cases were only detected by CT perfusion imaging, 8 cases were only detected by CT angiography, and the remaining 12 cases were diagnosed by CT perfusion imaging and CT angiography. Then, according to the diagnosis results of the CT image of the patients with cerebrovascular disease, these samples were followed up after 3 months, 6 months, and 9 months, and more accurate diagnosis results were obtained. The study showed that, after 3 months of CT detection, the sensitivity of patients with CTP detection was 67%, that of patients with CTA detection was 72%, and that of patients with combined detection was 83%. After 6 months of CT detection, the sensitivity of patients with CTP detection was 75%, that of patients with CTA detection was 79%, and that of patients with combined detection was 93%. After 9 months of CT detection, the sensitivity of patients with CTP detection was 86%, that of patients with CTA detection was 89%, and that of patients with combined detection was 99%. Therefore, the use of CTA combined with CTP joint detection of acute cerebrovascular disease imaging technology can effectively improve the diagnostic accuracy of patients.

## 1. Introduction

At present, the surgical technology and facilities of acute cerebrovascular disease have been greatly improved. Autologous tissue reconstruction of acute cerebrovascular disease is favored by more and more patients and surgeons, especially the continuous progress of imaging technology, which makes autologous tissue transplantation for breast reconstruction safer and more satisfactory [1]. The key to acute cerebrovascular disease is choosing the best perforator and vascular stalk. A three-dimensional reconstruction of the abdominal anatomical image after a CT scan gives the number and location of abdominal perforations, the course of the rectus abdominis muscle, and its distribution in the subcutaneous tissue.

In medical imaging research, Koshima et al. used chemical methods such as endothelial specific gene overexpression and fluorescent immunohistochemistry to study the role of cerebrovascular protein in the formation of atherosclerosis in adult patients and showed that cerebrovascular protein aggravated the damage of atherosclerotic endothelial cells by activating nitrosative stress and NLRP3 inflammatory bodies [2]. Allen and Treece proposed that *G βγ* subunits can directly bind and activate downstream effectors and start the *G* protein image transduction pathway of cerebrovascular proteins [3]. Minqiang et al. found that the upregulation of CVP gene in blood vessels helps to limit vascular leakage caused by VEGF and other vascular derived permeability factors [4]. Granzow et al. studied the role of cerebrovascular protein in angiogenesis and found that silencing cerebrovascular protein can reduce VEGF-induced VEGFR2, FAK, and Src phosphorylation and significantly reduce the expression of VEGF and VEGFR2, thereby reducing angiogenesis, suggesting that cerebrovascular protein may regulate VEGF/VEGFR imaging in angiogenesis [5].

In cell and vascular imaging, Wu et al. intercepted the extracellular domain (GCPF) containing RGD sequence of brain protein and evaluated whether the domain could target integrins *αvβ* 3 to improve the cognitive function of vascular dementia [6]. In vitro and in vitro vascular experiments of Voigt and Goerttler showed that GCPF had the biological activity of promoting angiogenesis, stimulating cell migration and adhesion, and promoting the growth of vascular endothelial cells [7]. Rozen et al. studied the role of cerebrovascular protein in the polarization and migration of pericytes and proved that cerebrovascular protein is highly expressed in pericytes and participates in the formation of filopodia through mediating cytoskeleton rearrangement [8]. Zhou Limei proposes timely diagnosis for patients with acute cerebrovascular disease with consciousness disorder, and provides active, reasonable and effective diagnosis and treatment to improve the treatment effect, which is conducive to the recovery of the patient's neurological function [9]. Rosson et al. study showed that the sensitivity, specificity, positive predictive value, and negative predictive value of high perfusion + uneven perfusion in the diagnosis of acute cerebrovascular disease were 48.00%, 91.89%, 92.31%, and 46.58%, respectively [10]. Masia et al. reported that the detection rate of “pseudocapsule sign” in acute cerebrovascular disease was 76.7%. In this group of data, the focus of acute cerebrovascular disease was small, and the maximum diameter was (31.34 4 ± 26) mm, and the detection rate of “pseudocapsule sign” was relatively low [11]. The above studies mainly focus on the diagnostic value of one or more typical symptoms, and the diagnostic rate of cerebrovascular disease is low. Therefore, this study analyzed and summarized all possible CEUS signs in clinical studies to better guide clinical applications.

CT perfusion imaging (CTP) and CT angiography (CTA) were used to diagnose cerebrovascular diseases. In this paper, 26 cases of patients with acute cerebrovascular disease in our hospital from June to August 2020 were selected as the research objects. According to the diagnosis method voluntarily chosen by patients, 6 cases were only detected by CT perfusion imaging, 8 cases were only detected by CT angiography, and the remaining 12 cases were diagnosed by CT perfusion imaging and CT angiography. Then according to the CT image of patients with cerebrovascular disease status of disease degree diagnosis, in 3, 6, 9 months of these samples for follow-up, and get more accurate diagnosis results.

## 2. Correlation Method between CT Imaging and Vascular Imaging

### 2.1. CT Perfusion Imaging and CT Angiography

#### 2.1.1. CT Perfusion Imaging

CT perfusion imaging (CTP) technology is a kind of noninvasive imaging technology with depth resolution, high resolution, and low cost, which has important application prospects in biomedical field [12]. Compared with the CTP image of static tissue, the CTP image of blood vessel shows more fluctuation, so optical coherence tomography (CTP) technology is developed. CTP needs to repeat A-scan or B-scan to record the change of spectrum image [13]. Commonly used CTP include speckle variance CTP and improved speckle contrast CTP imaging of vascular network in vivo [14]. However, limited by the imaging speed, the sample motion is an important source of motion artifacts (fringe noise) in the top view of CTP. The tissue motion is caused by the inevitable pulsation, breathing, and random motion of the sample blood flow [15]. The positioning accuracy of the galvanometer and the mechanical vibration of the system will also lead to motion artifacts. If the scanning speed of the galvanometer is unstable, the image intensity will weaken, and the image column will suddenly become bright or dark, showing bright or dark lines [16, 17]. Various factors may randomly affect the imaging process, resulting in the emergence of motion artifacts [18]. Motion artifact is shown as horizontal or vertical white line (stripe noise) in the top view of CTP, which seriously affects the visual quality of the image and is not conducive to its subsequent processing, such as image segmentation, classification, and disease diagnosis [19]. In the past few years, some methods have been developed in the field of CTP to suppress motion artifacts [20, 21]. Complex hardware is usually used to track the movement of the sample to guide CTP scanning [22]. In CEF algorithm, singular value decomposition is used to decompose the top view image into the first feature image containing motion artifacts and partial vascular features and the high pass feature image containing most vascular information [23]. Furthermore, the reconstructed first singular vector proposed in this paper is used to form the reconstructed first feature image in the form of outer product, so that the first feature image is further decomposed into two parts: the reconstructed first feature image (mainly including motion artifacts) and its orthogonal compensation product [24]. High pass feature image and orthogonal compensation product are used to reconstruct the restored image without motion artifacts. The experimental results verify the effectiveness of CEF algorithm, and the processed CTP top view has high image contrast. CEF algorithm makes up for the shortcomings of the traditional feature image filtering algorithm, which directly discards the first feature image algorithm and makes the image processed by the feature image filtering algorithm have higher signal-to-noise ratio and image contrast, which provides a new solution for removing similar fringe noise in the scanning system [25].

#### 2.1.2. CT Angiography

Orthogonal scanning or Lissajous scanning mode can be used to correct motion artifacts. However, these methods require additional equipment or improved scanning mode, resulting in additional costs [26]. In addition, motion compensation can reduce motion artifacts to a certain extent. 2D and 3D labeling methods reduce motion artifacts by splicing and reconstructing CTA images, but these labeling algorithms need large overlapping areas [27]. Tensor voting method is also used to correct the motion artifacts of CTA top view image. This method first segments the blood vessels and then fills the broken microvessels. However, if the fringe artifacts appear on the surface of the blood vessels, the fringe noise on the blood vessels still exists [28]. Similarly, removing motion artifacts based on the Bayes classification algorithm is prone to misjudgment. Microvessels are considered noisy and require a manually denoised B-frame image as a standard reference image. Frequency domain notch filtering algorithms (FRFs) have also been proposed to suppress the motion artifacts of the top view fringes of phase angiography CTA, but the image details are easy to be deleted together with the fringes, resulting in the loss of information of microvascular network [29]. These algorithms ignore the high linear correlation of fringe noise in the image [30, 31]. If the fringe and blood vessels can be mapped to different spaces according to the high linear correlation between stripes by some transformation or decomposition method, the image of useful blood vessels can be separated [32]. Therefore, this paper proposes a compensation feature image filtering (CEF) algorithm to remove the motion artifacts of CTA top view image. The feature image filtering algorithm based on singular value decomposition (SVD) is more widely used in seismic data processing [33, 34]. The random noise is suppressed by retaining the first few feature images, because the first few feature images contain highly correlated energy. At the same time, if the highly correlated energy is removed, the traditional feature image filtering algorithm will discard the first feature image and retain the high pass feature image to remove the fringe noise. In the top view of CTA, the linear correlation between the stripes of each row or column is very high, but the linear correlation between the stripes and blood vessels is low. If the top view of CTA is regarded as the superposition of a low rank matrix (fringe noise) and a high rank matrix (vascular feature), and the singular value decomposition can decompose the image into a series of characteristic images with rank 1, the fringe noise and vascular feature can be separated to a certain extent according to this characteristic. However, singular value decomposition (SVD) naturally decomposes the image into a grid-like feature image with rank 1 and linear correlation in both directions, and the fringes are only distributed in one direction. Therefore, it is necessary to improve the traditional feature image filtering algorithm.

### 2.2. CT Diagnosis of Acute Cerebrovascular Disease

CT is of great value in the diagnosis of acute cerebrovascular diseases in the skull base, which can clearly reproduce the types of acute cerebrovascular diseases. In addition, if acute cerebrovascular diseases and contusions in different parts of the skull are involved, the number of blows suffered by patients can be determined by CT scanning. It is also helpful to reduce the type of trauma by measuring the shape and size of acute cerebrovascular disease of skull with CT. In this case, the brain contusion caused by acceleration injury was mostly located at the impact site; the contusion of cerebral vascular injury is mostly located in the contraposition. Because the internal surface of occipital bone is smooth and the tentorial membrane structure of cerebellum has buffering effect, and the structure of skull base is uneven, the latest explanation for the contrecoup injury caused by hitting the frontal part is that, during collision, cerebrospinal fluid flows to the impact site to buffer the brain, while the opposite side of the impact point weakens the buffering effect due to the reduction of cerebrospinal fluid, so contrecoup brain contusion occurs. For acute extradural hematoma and subdural hematoma, acceleration injury is more likely to cause acute extradural hematoma than deceleration injury and more likely to occur in the same side of the impact site, often accompanied by acute cerebrovascular disease of skull. For subdural hematoma, cerebral vascular injury is more likely to cause subdural hematoma and more likely to occur in the opposite side of the impact site. It has been suggested that subdural hematoma may be associated with the detachment of cross-linked veins due to rotational movement. Sample selection is a typical case of linear motion brain injury and requires further analysis in the case of complex road accidents involving acceleration/deceleration processes or rotational shear force injury. CT images can accurately diagnose the type of craniocerebral trauma, provide timely and accurate image data for craniocerebral trauma, and be used as the preferred examination method for craniocerebral trauma. In addition, some studies believe that the impact site and stress propagation process can be reproduced by CT image data. This plays an important role in the cases of craniocerebral injury in forensic practice.

#### 2.2.1. Auxiliary Methods of CT Scanning System

Injury analysis is the establishment of craniocerebral injury graphic database, recording the patient's gender, age, injury location, injury mode, craniocerebral injury, and so on. CT images were mediated by frizzled family receptor and LRP5/6 through plasma membrane. Brain vascular protein imaging transduction complex specifically acts on *W* angiogenesis in endothelial cells of central nervous system.

(1) $$\begin{array}{c} W_{1}=\left\{\begin{array}{c} s-p_{1}-x_{1},\\ x-p_{2}-\left(1-x_{1}\right), \end{array}\right.\\ \text{FZD}{}_{1}=\frac{p_{2}-p_{1}+1}{2}. \end{array}$$

Conventional ultrasound is the basis of all new ultrasound technology applications, and contrast-enhanced ultrasound makes up for the shortcomings of conventional ultrasound in detecting small vessels and low-speed blood flow *P*:

(2) $$\begin{array}{c} p_{1}^{*}=\frac{2k}{k+1}+\frac{2c_{1}+c_{2}+3et+2\text{RAML }\zeta }{3},\\ \frac{\partial \pi_{A}^{\text{LH}}}{\partial p_{1}}=\frac{p_{2}-p_{1}+1}{2}-\frac{p_{1}-c_{1}}{2}+\frac{p_{2}-p_{1}+k}{2k}-\sum_{x=1}^{13}Vx-e\left(1-\zeta \right)t\left[-\frac{1}{2}-\frac{1}{2k}\right]\\ =0. \end{array}$$

Compared with contrast-enhanced CT or MRI, contrast-enhanced ultrasound is easy to operate, has no radiation damage, can continuously observe the microcirculation perfusion in real time, can be repeatedly checked if necessary, and has a better clinical application prospect. SonoVue is a pure blood pool contrast agent, which is mainly discharged through the lung, and has no toxicity to liver, kidney, and heart.

(3) $$\begin{array}{c} V=\sum_{x=1}^{13}Vx\\ =\sum_{x=1}^{13}\left(\frac{Wx}{\sum_{1}^{n}W13}Sx\right). \end{array}$$

Especially when gray-scale ultrasound showed hyperechoic features and contrast-enhanced ultrasound showed fast-forward, high perfusion, uneven perfusion features with or without ring enhancement, RAML could be basically excluded to make the diagnosis of acute vascular disease.

(4) $$\begin{array}{c} {\text{CT}}_{2}^{*}=\frac{2k}{k+1}+\frac{c_{1}+2c_{2}+3et-3et\zeta }{3}. \end{array}$$

Avoid delaying clinical treatment. It is suggested that close follow-up or CT or MRI examination should be combined to avoid over treatment.

(5) $$\begin{array}{c} {\text{RAML}}_{1}=\frac{p_{2}-p_{1}+1}{2}. \end{array}$$

It is closely related to ischemic stroke, atherosclerosis (as), hypertension, multiple sclerosis, and cancer. Therefore, in-depth study of the physiological and pharmacological functions of cerebrovascular proteins is expected to provide new therapeutic targets for these diseases. In this review, we will summarize the known functional characteristics of cerebrovascular proteins, introduce their main research progress in physiology and pharmacology, and focus on the image transduction B and related pathway *W*: 1, which interact with cardiovascular and cerebrovascular diseases.

(6) $$\begin{array}{c} w_{ik}=\sum_{a}^{n}\tau_{1}X_{ik}+\sum_{b}^{n}\tau_{2}U\left(Y_{ik}\right)+B_{ik}. \end{array}$$

#### 2.2.2. Association Algorithm of Cerebrovascular Protein and Biological Characteristics

Cerebrovascular proteins are a large family of proteins, which transmit a variety of physical and chemical images, including neurotransmitters, hormones, growth factors, and aromatics. Cerebrovascular protein superfamily is composed of about 800 receptors. Based on amino acid sequence similarity and common physiological characteristics, it can be divided into five subfamilies: the largest is rhodopsin family, which has about 284 members in humans, followed by adhesion family with 33 members, followed by glutamate family, secret family, and frizzled family. At the tissue level, the CVP expression is different between normal people and patients. The expression of CVP was low in human heart, placenta, and small intestine, but also in liver, kidney, pancreas, and spleen. Expression of CVP was detected only in the brain, heart, lungs, skeletal muscle, pancreas, and intestine, not in the human brain, thymus, adrenal gland, renal cortex, spinal cord, liver, spleen, or stomach. At the cellular level, cerebrovascular proteins are widely expressed in endothelial cells of various tissues, including brain, heart, retina, kidney, and pancreas, which indicates that cerebrovascular proteins may be related to angiogenesis, arteriosclerosis, and other physiological processes. As a member of adhesion family, cerebrovascular proteins have the typical structural characteristics of this family as *C*(*t*):

(7) $$\begin{array}{c} c_{1}\left(t\right)\geq 0\text{,}\\ c_{2}\left(k\right)\geq 0\text{,}\\ c_{3}\left(k\right)\geq 0\text{,}\\ c_{4}\left(k\right)\geq 0\text{,}\\ c_{5}\left(k\right)\geq 0. \end{array}$$

However, there are some limitations in the diagnosis of lesions, which need to be combined with enhanced examination. RAML is the most common benign renal vessel. Generally, follow-up observation is enough. When the tumor is large or accompanied with bleeding, nephrectomy can be performed. It has been reported that renal cell carcinoma accounts for a large part of acute renal vascular disease. The clinical treatment strategy LH is local resection or radical nephrectomy:

(8) $$\begin{array}{c} \pi_{B}^{\text{LH}}=\frac{2k}{k+1}+\left[\frac{1}{2}+\frac{1}{2k}\right]{\left[\frac{c_{1}-c_{2}}{3}\right]}^{2}+\frac{2\left(c_{1}-c_{2}\right)}{3}. \end{array}$$

How to effectively improve the accuracy of renal vascular diagnosis to promote clinical precision treatment is a problem worthy of attention. It is reported that hypoechoic mass with rich blood supply is common in acute cerebrovascular disease, and hyperechoic mass with poor blood supply is common in RAML. However, studies have shown that hyperechoic cerebral vessels are not uncommon, and the conventional ultrasound manifestations of atypical cases often overlap. Hyperechoic cerebral vessels and hypoechoic RAML are the difficulties in ultrasonic differential diagnosis. Among them, adhesion family has attracted much attention due to its unique structure, except for 7TM *α*. In addition to the helical transmembrane domains, they also have a large number of conserved extracellular N-terminal domains and a proteolysis inducing domain of cerebrovascular proteins. Cerebrovascular protein is one of the three membrane receptors of transmembrane image transmission, which is distributed in almost all tissues and organs.

## 3. Experimental Design of CT Imaging Combined Diagnosis

### 3.1. Research Methods

CT perfusion imaging and CT angiography were used to diagnose cerebrovascular diseases. In this paper, 26 cases of patients with acute cerebrovascular disease in our hospital from June to August 2020 were selected as the research objects. According to the diagnosis method voluntarily chosen by patients, 6 cases were only detected by CT perfusion imaging, 8 cases were only detected by CT angiography, and the remaining 12 cases were diagnosed by CT perfusion imaging and CT angiography. Then according to the CT image of patients with cerebrovascular disease status of disease degree diagnosis, in 3, 6, 9 months of these samples for follow-up, and get more accurate diagnosis results.

### 3.2. Inspection Methods and Contents

The size of the blood vessels was measured, and the echo, boundary, and color blood flow image of the blood vessels were observed. The blood vessels were divided into hypoechoic group (including hypoechoic, cystic, and solid mixed echo with hypoechoic solid components) and nonhypoechoic group (including hyperechoic, isoechoic, mixed echo with hypoechoic solid components). The solid component was mixed cystic and solid echo with high or equal echo. Then, the best section which can clearly show the blood vessels and the surrounding renal parenchyma was selected as the contrast observation section. The patient was asked to breathe calmly and slowly, and the low mechanical index mode was selected. The contrast medium was injected through the superficial vein of elbow (0.8–1.0 ml each time) and 5 ml physiological saline was added. At the same time, the timekeeping button was pressed and the entire process was recorded on the HD hard disk. Otherwise, it was “slow regression” perfusion intensity (the peak intensity of contrast medium perfusion being higher than or equal to the surrounding renal cortex is called “high perfusion”; otherwise, it is “low perfusion”), perfusion uniformity, and peripheral annular enhancement.

In the diagnosis, statistical methods were used to analyze the diagnostic rate of different CT methods. Cerebrovascular proteins not only participate in the basic pathophysiological processes such as angiogenesis, maintenance of blood-brain barrier function, and endothelial inflammatory response but also can be used as potential drug targets for the treatment of cardiovascular and cerebrovascular diseases and their complications. At present, the known experiments and studies on cerebrovascular proteins are based on animal models, but the specific mechanism of action in human tissues and organs has not been clarified. There are still many problems to be solved, including the ligand identification, activity detection, and the mechanism of important image transduction pathways.

## 4. Results and Discussion

### 4.1. Diagnostic Ability of  CT Imaging in Acute Cerebrovascular Disease

As shown in Figure 1, 53.41% of acute cerebrovascular diseases and 31.58% of RAML had blood flow images. Hyperechoic acute cerebrovascular diseases and hypoechoic RAML accounted for 12.50% and 13.16%, respectively. The pathological type of the latter was less fat. Conventional ultrasound combined with contrast-enhanced ultrasound is helpful in the differential diagnosis of acute cerebrovascular disease and RAML, but the value of contrast agent perfusion intensity in the differential diagnosis of benign and acute renal vessels is controversial. Some scholars believe that there is no significant difference in perfusion intensity between cerebral vessels and RAML after contrast-enhanced ultrasound. Others believe that the perfusion intensity of renal benign vessels is significantly lower than that of renal acute vessels. Others believe that the perfusion intensity of acute cerebrovascular disease is related to the size of lesions. The larger the lesions, the higher the perfusion intensity. The data showed that hyperperfusion was an effective index in the differential diagnosis of acute cerebrovascular disease and RAML, with high accuracy, sensitivity, and positive predictive value.

As shown in Figure 2, the lesions of acute cerebrovascular disease had mainly low echo level, rich blood supply, and clear boundary, while the lesions of RAML had mainly non-low echo level, lack of blood supply, and clear boundary. There were significant differences in echo level and blood supply distribution between the two groups. Taking rich blood supply as the diagnostic standard of acute cerebrovascular disease and lack of blood supply as the diagnostic standard of RAML, the value of conventional ultrasound in differential diagnosis of ccRCC and RAML lesions in low echo group and non-low echo group was analyzed. The results are shown in Table 1. The specificity and positive predictive value of conventional ultrasound in differential diagnosis of acute cerebrovascular disease and RAML lesions in low echo group are higher.

As shown in Table 1, when the frontal part was impacted, the corresponding part of the cerebral vascular injury occurred. When the temporal part was impacted, there were 14 cases of cerebrovascular injury, 5 cases of contralateral contrecoup injury, and 1 case of cerebrovascular injury, contrecoup injury, compound injury. When the parietal lobe was impacted, there were 10 cases of cerebral vascular injury in parietal lobe, less cerebral vascular injury, contrecoup injury. When the occipital part was impacted, it was more prone to be hit, and there are fewer cases of combined damage and cerebrovascular damage caused by impact. Among the cerebral vascular injuries, 21 cases of cerebral vascular injuries were located at the landing site, and 26 cases of cerebral contrecoup injury were located at the opposite side of the landing site. There were 12 cases of cerebral vascular injury, 1 case of contrecoup injury, and 7 cases of impact contrecoup injury.

As shown in Table 2, of the 22 cases of cerebrovascular injury, 18 cases were prone to occur on the side of external force impact, and 4 cases were located on the opposite side of impact. For subdural hematoma, cerebrovascular injury was more likely to occur than acceleration injury, accounting for 14.08% and 12.20%, respectively. There were 21 cases of subdural hematoma on the contralateral side, and 18 cases on the side of impact site. Among 23 cases of accelerated injury, 12 cases were located in the contralateral area and 7 cases in the ipsilateral area. For subarachnoid hemorrhage, the main location of subarachnoid hemorrhage is at the base of brain tissue and the side fissure cistern and sulcus of brain contusion area.

As shown in Figure 3, vessels with fast-forward signs in CEUS-related diagnostic indicators tend to be acute. The accuracy, sensitivity, positive predictive value, and negative predictive value of differential diagnosis of acute cerebrovascular disease and RAML are high, and the probability difference of fast-forward signs between acute cerebrovascular disease and RAML lesions is statistically significant. Analysis of the possible causes is that the number of new blood vessels in acute vessels is large, the inner diameter is large, and arteriovenous fistula is formed after destroying normal vessels, which makes the focus rich in blood supply, so the perfusion speed of contrast medium is fast, the degree is high, the duration is short, and the regression is fast. The pathological basis for slow perfusion rates and low perfusion intensities in contrast-enhanced ultrasound may be the lack of vascular components, narrow lumens, and elastic layers. Repeated circulation of microbubbles in a winding microvascular network may be the reason for the delay in contrast media.

As shown in Figure 4, the pathological basis of “pseudocapsule sign” is annular enhancement around cerebral vessels, but vascular cells can infiltrate and break through the pseudocapsule into normal renal tissue. In this group of data, 10.53% of RAML showed ring enhancement, and 34.09% of acute cerebrovascular disease showed ring enhancement, of which 2 cases were incomplete. The specificity and positive predictive value of peripheral ring enhancement sign in the differential diagnosis of acute cerebrovascular disease and RAML were higher, but the sensitivity was lower. The difference of peripheral ring enhancement rate between the two groups was also statistically significant.

As shown in Figure 5, during angiogenesis, VEGF mainly emits images through VEGFR2 and activates downstream factors such as SRC, FAK, Akt, ERK, and JNK, thus regulating the proliferation, migration, and invasion of endothelial cells.

As shown in Table 3, CT imaging and its coreceptor neuropilin-1 play an important role in cerebral angiogenesis and blood-brain barrier differentiation. In the process of embryonic development, the analysis of VEGF expression in cerebral vascular proteins showed that VEGF164 was the main expression form, while vegf120 and vegf188 had low expression levels, but each VEGF variant was overexpressed in the brain. Therefore, the knockout of CVP may lead to the upregulation of VEGF, cause vascular leakage, and affect the formation of blood-brain barrier.

As shown in Figure 6, the embryonic death caused by cerebrovascular protein is due to the stagnation and hemorrhage of angiogenesis in the central nervous system, while the overexpression of blood vessels leads to the abnormal proliferation of blood vessels in the central nervous system, which indicates that cerebrovascular protein is related to the vascular pathology of various central nervous system diseases.

As shown in Figure 7, there were 3 cases of cerebral vascular injury when the top touched the ground. There were 1 case of cerebral vascular injury, 14 cases of cerebral contrecoup injury, and 2 cases of impact contrecoup injury. The frontal lobe and cerebrovascular accidents are the most common sites of direct intracerebral injuries, and the occipital region has the highest incidence of direct intracerebral injuries. Direct injuries often occur in the bilateral frontal lobes and cerebrovascular accidents. For acute epidural hematoma, accelerated injury was more likely to occur than cerebrovascular injury, accounting for 14.33% and 7.94%, respectively. Acute epidural hematoma often occurs at the site of external force impact, such as accelerated brain injury, and 20 cases of acute epidural hematoma, 12 cases in the same side of the impact, 6 cases in the opposite side of the impact have occurred.

As shown in Figure 8, it may be because the action of lateral strike conforms to the habit of people waving objects and the resistance is small. In daily life, the striking force is big in the common fighting events. The different ways of injury and the different types of head injury will affect the distribution of craniocerebral injury and thus affect the judgment of craniocerebral injury. This study found that different types of craniocerebral injury were caused by different ways of injury: scalp injury, acute cerebrovascular disease of skull, that is, the injury was mainly concentrated on the outside of the impacted brain, and often multiple strikes, resulting in multiple parts of the injury.

As shown in Table 4, the main types of injury in cerebrovascular injury are subarachnoid hemorrhage, scalp injury, and brain contusion, and the injury is mainly intracranial. Among them, the typical deceleration craniocerebral injuries such as flat fall and high fall are mainly brain contusion. In addition, by comparing the types of cerebral contusion, it is found that, in accelerated injury, cerebrovascular injury is often caused. In deceleration injury, the common type of brain contusion is contrecoup injury.

As shown in Figure 9, among the four contrast-enhanced ultrasound signs in the differential diagnosis of acute cerebrovascular disease and RAML, the high perfusion accuracy is the highest, the ring enhancement specificity is the highest, the fast-forward sensitivity and negative predictive value are the highest, and the positive predictive value of uneven perfusion is the highest. When combined with the two diagnostic indicators for differential diagnosis, the accuracy and sensitivity of fast-forward + high perfusion are higher, which can effectively improve the diagnostic accuracy of acute cerebrovascular disease and reduce the rate of missed diagnosis.

After 3 months of CT detection, as shown in Figure 10, the sensitivity of patients with CTP detection was 67%, that of patients with CTA detection was 72%, and that of patients with combined detection was 83%. After 6 months of CT detection, the sensitivity of patients with CTP detection was 75%, that of patients with CTA detection was 79%, and that of patients with combined detection was 93%. After 9 months of CT detection, the sensitivity of patients with CTP detection was 86%, that of patients with CTA detection was 89%, and that of patients with combined detection was 99%.

### 4.2. Discussion

There are different ways of injury and types of craniocerebral injury distribution, and the vast majority of craniocerebral injury can be related to the scalp, so for cases of craniocerebral injury, CT images can be used to evaluate the impact site of the injury. For the two types of scalp injury, the detection rate of CT is not high, so it is necessary to refer to the results of forensic clinical examination when judging the scalp injury. The type of skull acute cerebrovascular disease can help to determine the location and nature of external force. Its location and direction are consistent with the trend of acute cerebrovascular disease. In the study of blow injury, 6 cases of acute cerebrovascular disease of skull base were found to have suffered frontal blow. The reason of acute cerebrovascular disease of skull base may be that when the frontal part was impacted, the line of acute cerebrovascular disease turned to the anterior skull base. Among the 3 cases of acute cerebrovascular disease of skull base caused by falls, 2 cases of acute cerebrovascular disease of sphenoid bone in middle cranial fossa were caused by temporal stress, and 1 case of acute cerebrovascular disease of orbital plate in anterior cranial fossa was caused by frontal stress. The reason may be that the stress is transmitted to the weak anterior skull base through the skull due to the impact on the occipital and parietal parts.

CT transverse scan can show scalp hematoma, brain contusion, and laceration intuitively and clearly, so it is of great significance for the diagnosis of craniocerebral trauma. The main problem that forensic professionals need to solve is to distinguish whether the head injury is due to a blow or a fall by analyzing the injury mode. Currently, more than 36% of the drugs on the market target cerebrovascular protein, the most popular drug target. Therefore, mastering the regulatory mechanism of cerebrovascular proteins is a key step in the development of new drugs, which can also play an important role in the prevention and treatment of related diseases. In the vascular system, there is a lack of expression of cerebrovascular protein, and the embryo shows delayed neural tube vascular invasion, developmental defects, and hemorrhage. TGF-*β* gene deletion in the pathway will lead to abnormal angiogenesis in the forebrain and spinal cord of the patient embryo, which is similar to the vascular phenotype seen in the deletion mutants of CVP.

## 5. Conclusions

In patients with acute cerebrovascular disease, the abnormal distribution and deposition of collagen and the abnormal aggregation of smooth muscle cells were observed by immunohistochemistry. Stimulating TGF-*β* can specifically cause the formation of basement membrane and the recruitment or differentiation of smooth muscle cells, which further proves that the lack of cerebrovascular protein in blood vessels will lead to TGF-*β.* The image was elevated. The relationship between cerebrovascular protein and TGF-*β* image pathways can build a potential model. Therefore, cerebrovascular protein can affect the occurrence and development of atherosclerosis by inhibiting the activation of NLRP3, which can be used as a potential drug target for the prevention and treatment of atherosclerosis in the future. In this study, we found that the expression of CVP was upregulated during the dedifferentiation of skeletal muscle smooth muscle cells and negatively regulated the expression of inflammatory factors in skeletal muscle smooth muscle cells, suggesting that CVP may be a potential target for regulating blood pressure. The role of CVP in the development and development of hypertension has been studied. We found that CVP is expressed in the aorta, heart, kidneys, and brain. However, in hypertension, CVP expression is upregulated in the left atrium and left ventricle. This indicates that overexpression of CVP can increase angiogenesis and reduce myocardial damage caused by hypertension. Further studies on the pathophysiological mechanism of CVP, its role in cardiovascular and cerebrovascular diseases, and its possibility as a drug target have a good application prospect. However, due to the lack of known agonists/antagonists and the lack of data on their role in the regulation of vascular tension or other smooth muscle cell functions, whether cerebrovascular proteins are involved in the regulation of blood pressure remains to be further studied.

## Figures and Tables

**Figure 1:** Perfusion intensity difference after contrast-enhanced ultrasound.

**Figure 2:** CT perfusion imaging of acute cerebrovascular disease.

**Figure 3:** Fast-forward signs of blood vessels during CT imaging.

**Figure 4:** Circle around the cerebral blood vessels.

**Figure 5:** Image processing during dynamic imaging.

**Figure 6:** Central nervous system angiogenesis stagnation and bleeding.

**Figure 7:** The most common part of brain hedging injury.

**Figure 8:** Different ways of injury and types of head injury.

**Figure 9:** Contrast-enhanced ultrasound signs in acute cerebrovascular disease.

**Figure 10:** The sensitivity of patients undergoing joint testing.

**Table 1:** Cerebral vascular impact injury after contrast-enhanced ultrasound perfusion intensity.

Item	ccRCC	Lack of blood supply	Tube wall	Low echo	Boundary
Identify	1.21	1.83	2.91	3	3.61
Forecast	2.86	5.88	5.48	2.73	3.46
Average	2.97	1.43	1.87	2.63	5.7
Training error	2.77	1.05	3.63	2.39	4.98
Test error	3.44	2.42	3.4	3.42	1.01

**Table 2:** Contrast-enhanced ultrasound site brain impact injury.

Item	Lesion	Contrast agent	Blood supply	Tube wall	Boundary
Test error	1.3	0.35	1.75	1.15	0.24
Angiography	2.06	3.44	2.31	2.4	1.16
Perfusion intensity	2.53	5	3.64	3.02	3.56
Cerebrovascular injury	2.02	1.75	5.93	3.72	5.49
Lesion	3.86	2.17	4.74	4.42	4.62

**Table 3:** Cerebral angiogenesis and blood-brain barrier differentiation.

Item	Blood supply	Tube wall	Low echo	Boundary	Venous fistula
Training error	3.92	1.08	3.59	3.8	3.59
Test error	5.3	4.95	5.89	3.51	2.99
Angiography	3.23	1.17	5.51	3.39	4.57
Perfusion intensity	4.39	2.45	1.42	4.19	3.35
Cerebrovascular	3.9	6.15	4.07	6	4.05

**Table 4:** Types of deceleration head injury and brain contusion.

Item	Contrast agent	ccRCC	Blood supply	Tube wall	Low echo	Boundary
Blood flow	1.79	0.82	0.35	0.51	0.5	6.43
RAML	1.9	3.14	2.02	1.22	1.19	6.88
Identify	3.73	4.9	3.61	2.74	4.75	2.44
Forecast	1.02	5.54	2.51	3.3	4.08	1.08
Average	1.29	3.15	1.19	1.12	4.7	3.21
Training error	5.35	5.21	5.47	6.51	6.29	2.66

## Data Availability

The data that support the findings of this study are available from the corresponding author upon reasonable request.
